RETRACTED

# Optimal Modeling and Simulation of the Relationship between Athletes' High-Intensity Training and Sports Injuries

**DOI:** 10.1155/2022/8447453

**Published:** 2022-09-14

**Authors:** Youcheng Zhang, Yuanyuan Chang

**Affiliations:** College of Physical Education, Taiyuan University of Technology, Jinzhong, Shanxi 030600, China

## Abstract

In order to take into account the physical health of athletes and the quality of sports training, an optimization modeling and simulation method for the relationship between high-intensity training and sports injuries of athletes is proposed. The research of the specific content of the method is based on the two-dimensional and three-dimensional registration principles. In the research process, the program is written strictly according to the registration principle, and the correctness of the method is effectively tested by means of experimental methods. Digital image reconstruction measures based on 3D models may be based on ray tracing methods. The experimental results show that the number of accurate cases of this method is 77, and the accuracy rate is 96.3%. The proposed method can formulate a scientific and effective injury prevention strategy for athletes during high-intensity training.

## 1. Introduction

With the development of sports, the industry is paying more and more attention to sports injuries. It is believed that sports injuries mainly refer to the results that occur in the process of training and competition, resulting in the reduction of the athlete's athletic ability, which can only be recovered through treatment, or the result of the athlete's poor social ability. It is believed that the research on sports injury should move from analysis to integration. Sports injury is an abnormal physical injury phenomenon that occurs in the process of sports training preparation activities or formally participating in sports [1]. The injury is affected by its own physiological condition, external environment, and sports characteristics. Sports injuries here are distinguished from accidental bodily injuries in daily life, which are highlighted by the inevitable relationship between the injury and the skills required to perform a certain sport.

The development of sports training can not only improve the physical quality of young athletes but also improve the psychological quality of young athletes. This means that physical training is of great significance to the development of young athletes. However, in the process of sports training, sports injuries are very likely to occur, and sports injuries not only affect the physical health of young athletes but also cause huge psychological pressure on young athletes and may even affect the students and living conditions of young athletes; at the same time, it has a certain degree of impact on teachers' teaching tasks and teaching plans. Therefore, it is very necessary to prevent sports injuries in sports training of young athletes [2].

RETRACTED

Surveys show that more than 70% of the injuries suffered by athletes during training can be avoided. Prevention is fundamental to reducing physical harm. In the process of daily sports training, training teachers and athletes must learn the knowledge of scientific prevention of sports injuries, strengthen the awareness of self-protection of athletes, so as to effectively reduce or avoid sports injuries, reduce the negative impact of sports injuries, and maintain the physical and mental health of athletes, healthy, and athletes can effectively engage in daily sports training.

## 2. Literature Review

The internal factors that cause sports injuries in the sports training of young athletes mainly include the following points: first, lack of ideological awareness. Sports injuries occur in young athletes in sports training, mainly because teachers and young athletes have insufficient ideological understanding of the meaning of sports injuries, and teachers lack the awareness of sports injury prevention for young athletes and blindly carry out sports in sports training, eager for success, often causing acute joint injuries in young athletes. Second, physical training preparation activities are unreasonable. The preparatory activities before sports training are to change the young athletes' bodies from quiet to active state, if the preparatory activities for sports training are insufficient, the chances of sports injuries for young athletes will be greatly increased, if the preparatory activities are excessive, it will cause young athletes to be in a state of fatigue and no longer suitable for sports training, thus increasing the occurrence of sports injuries in sports training for young athletes. Third, young athletes have low physical fitness. The low physical quality of young athletes is the fundamental cause of sports injuries in sports training. No matter what kind of sports, young athletes are required to have certain physical qualities, such as track and field requires speed and endurance, shot put requires strength, and gymnastics requires flexibility[3]. If young athletes do not have the corresponding physical fitness to carry out sports training, it will cause sports injuries, and even if young athletes carry out sports training when they lack special qualities, the probability of sports injuries for young athletes will be higher.

Based on the above problems, the author proposes a method for sports medicine image modeling and injury prevention in the process of sports training. The specific content of this method is that, according to the research situation of medical image 3D modeling and registration technology for precise radiotherapy devices, the functions of the medical image navigation system can be enriched to enhance the accuracy of the model [4]. In order to shorten the modeling time, the complexity of 3D modeling can also be appropriately reduced according to the actual situation of the research work. During the study period, a retrospective analysis was carried out according to the patient's diagnosis; during the period, the experimental verification platform included X-ray machines, graphic workstations, operating beds, and other equipment. According to the actual situation of the experimental research, the relevant personnel used CT equipment to complete the scanning of bone information and input the relevant image data into the workstation, processing to determine the closed contour of each image in the CT data. The method used in the construction of the 3D model is the volume mapping algorithm [5]. During the construction of the 3D model, the relevant personnel used image noise reduction measures, remove noise in CT image data, and improve image quality. Use the image segmentation tool for image segmentation algorithms during modeling. During the implementation of the three-dimensional reconstruction of CT data, relevant personnel use surface rendering and volume rendering to realize the three-dimensional image surface.

RETRACTED

## 3. Method

### 3.1. Acquisition of Medical Images

Medical images are obtained by scanning the patient's lesions with various medical imaging equipment. With the development of science and technology, more and more new medical imaging devices are used in clinical practice. At present, the mainstream medical image acquisition methods are as follows: X-ray tomography (CT), magnetic resonance imaging (MRI), and positron emission tomography (PET) [6]. Each of these medical imaging devices has its own characteristics and advantages, but the principles of imaging are similar, and they all use Fourier transform or Radon inversion algorithms to infer three-dimensional space from ray projections in multiple directions, a certain physical property of an object in the system, and finally reconstruct the result to generate a tomographic image.

In order to unify the interface standards between equipment of different manufacturers and unify the image formats obtained by a variety of medical imaging equipment, the American College of Radiology (ACR) and the National Electrical Manufacturers Association (NEMA) formulated a unified standard in 1983, the standard storage format dedicated to medical images, the ACR-NEMA standard released in 1985. The Digital Imaging and Communications in Medicine (DICOM) 3.0 standard released in 1993 is the current international standard in the field of medical imaging informatics [7].

RETRACTED

DICOM file consists of two parts: file header information (DICOMFileMeta Information) and DICOM data set (DICOMDataSet) [8]. The file header contains the identification information of the dataset (FilmMetaInformation), including the file identification prefix, dataset identification, storage format, and patient medical information. The DICOM data set uses the data element (DataElement) as the coding unit, and each data element stores the value of a certain attribute in the data set, including the following parts: Tag (Tag), data type (VR), data length (ValueLength), and data Field (ValueField). Multiple data elements are aggregated together to form a dataset. The format of the DICOM file and the encoding format of the data elements are shown in Figure 1.

According to the structure of the DICOM file, the program can read the image information in the DICOM file and convert it into a three-dimensional space data field.

### 3.2. VTK Class Library

Visualization Toolkit (VTK) is an open-source system visualization toolkit developed by Corporate R&D, it is mainly used for the writing of 3D computer graphics, image processing, and visualization programs, and the field of application is quite extensive. Its core is built with C++ and contains about 250,000 lines of code, more than 2000 classes, and several conversion interfaces; so, VTK can be freely used in Java, Python, and other languages. VTK uses object-oriented technology to encapsulate common algorithms in the field of image visualization into classes, which enables programmers to directly call algorithms through interfaces.

In order to manage the huge class library inside VTK simply and effectively, the classes included in VTK are divided into common base class (Common), graphics operation class (Imaging), graphics algorithm class (Graphics), data format conversion class (Filtering), and graphics rendering class (Rendering), etc. and generate the corresponding dynamic link library. Among them, the common base class is the parent class, and the other classes are the inheritance of the common base class and complete their own work according to specific requirements [9]. In addition to the C++ class library, VTK comes with an interpretation packaging layer system to wrap the C++ class library, which is convenient for the use of languages such as TCL and Java. The advantage of using this architecture is that programmers can use the C++ language to create efficient algorithms, and other scripting languages can be used for rapid development.

RETRACTED

VTK uses data flow to convert source data into image data, this data exchange relationship is called Pipeline, which contains two basic objects: data object (vtkDataObject) and processing object (vtkProcessObject) [10]. The data object represents the data information such as the geometric structure, topological structure, and unit gray value of the image, and the processing object is also called the filter (Filter), which is used to manipulate and process the data object and generate new data. The processing object represents the algorithm by which the system processes the data. As shown in Figure 2 below, VTK connects data objects and processing objects through the data visualization pipeline to complete the data processing.

### 3.3. Image Preprocessing

#### 3.3.1. Removing Image Noise

Noise is a collection of pixel distortions caused by various reasons in the image generation process. The existence of noise may affect the diagnosis of tiny lesions by doctors and may even lead to misdiagnosis and delay the treatment of patients. Therefore, sufficient attention must be paid to noise.

Since CT images are easily disturbed by noise during transmission and acquisition, in order to improve the quality of the images as much as possible, the images must be denoised and smoothed [11]. At present, many methods of image denoising have been proposed, such as neighborhood averaging method, median filtering method, and Gaussian filtering algorithm; according to some characteristics of medical images, we choose a method that can remove noise well and also a denoising method to protect image edge information.

Because precise radiotherapy requires real-time positioning, and the data scale of each set of CT is relatively large, it puts forward requirements for image processing time.  Table 1 shows the processing time of three image filtering methods measured by computer for a single image.

It can be seen from Table 1 that the average neighborhood filtering method takes the least time and requires the least amount of computation, while the median filtering method takes the longest time and has the largest amount of computation [12]. The median filter method takes 2.29 times as long as it is the Gaussian low-pass filter method and 16 times as long as it is the average neighborhood method.

The denoising ability of median filtering and Gaussian low-pass filtering is weaker than that of average neighborhood filtering, but while removing noise, average neighborhood filtering will cause the image to deform locally at the boundary, which affects doctors' judgment of the disease [13]. Although the average neighborhood has the advantages of small calculation and short processing time, it cannot meet the requirements of retaining feature points on the boundary; so, it is not suitable for the imaging system of radiotherapy. To sum up, this subject chooses Gaussian low-pass filtering as a method to remove image noise.

RETRACTED

### 3.4. Establishment of 3D Model

Using the abovementioned methods of image denoising, threshold division, contour extraction, etc., the software system completed the preprocessing of CT images and obtained the closed contour of each image in the CT data set, which was carried out for the MC algorithm. 3D modeling is ready for work.

The 3D reconstruction technology extracts the corresponding data point set from the tomographic sequence image according to the set threshold to form the isosurface. According to the principle of triangulation, the isosurface is divided into several triangular patches, and the triangular patches are rendered by the graphics lighting model to form a three-dimensional image, so as to achieve the purpose of intuitive display of geometry. The program development kit of Visualization Toolkit (VTK) is widely used in the construction of 3D images. By calling the class library in VTK, the development of 3D software can be carried out quickly and efficiently, so that it has a powerful 3D graphics display function and can realize interactive 3D measurement.

Early three-dimensional modeling methods include Fourier transform and convolution back-projection. With the development of imagery, three-dimensional modeling methods such as multilevel reconstruction (MPR), maximum density projection (MIP), surface rendering, and volume rendering have been proposed [14]. The most widely used 3D modeling methods are surface fitting and Voxel-based volume rendering.

The basic steps to achieve 3D modeling with VTK are as follows:

1. Preprocessing of CT slice data: image denoising method is used to remove noise in CT image data and improve image quality
2. Segmentation of CT data: the CT image is segmented using an image segmentation algorithm, and the image edge dataset is searched
3. 3D reconstruction of CT data: according to the image edge data set, the surface rendering and volume rendering methods are used to realize the three-dimensionalization of the image surface. In this subject, the MC algorithm is used to realize the three-dimensional reconstruction of medical images

#### 3.4.1. Surface Reconstruction Algorithm and Volume Rendering Algorithm

The moving cube method (marching cubes, MC algorithm) is currently the most popular 3D reconstruction method [15]. The basic idea of the MC algorithm is as follows: according to the input tomographic image sequence, after segmentation and extraction, a three-dimensional data field is formed, the cubes intersecting with the isosurface are processed one by one, and then the intersection of the isosurface and the cube is calculated by the interpolation method. According to the relative position relationship between the intersection of the cube and the isosurface, connect the intersection of the isosurface and the cube in a certain way to form a new isosurface.

RETRACTED

Voxel-based volume rendering methods can generally be classified into image-order methods, object-order methods, and hybrid-order methods. The algorithm based on the image space sequence method is represented by the ray casting method proposed in 1988 [16]. The algorithms based on the object space order method mainly include the footprint method (SplattingAlgorithm or FootprintAlgorithm), the sputtering algorithm (Splatting), and the shear warp algorithm (ShearWarp). The algorithm based on the hybrid order method has the shearwarp factorization algorithm. The advantage of the volume rendering algorithm is that there is no need for segmentation, and the volume data can be directly rendered through the set transformation function.

### 3.5. Digital Image Reconstruction

#### 3.5.1. Principle of Digital Image Reconstruction

Digital image reconstruction (digitally reconstructed radiograph, DRR) is to generate a three-dimensional spatial data field from CT image data and observe the digital projection image obtained from any direction in the spatial data field [17]. In order to simulate a real X-ray image, the information that DRR needs to simulate includes characteristics such as attenuation and scattering of X-rays as they pass through the 3D spatial data field. By calculating the attenuation of each ray through three-dimensional space, a simulated projected image is obtained on film.

There are two methods to obtain DRR images: projection method and ray tracing method. The projection method is to project each voxel on the film position, and the brightness of the pixel is proportional to the density of the projected voxel to obtain an analog image. The ray tracing method is to trace the intersection of each ray emitted from the light source and each pixel in the three-dimensional model and accumulate the density of the voxels that each ray passes through. The brightness value of the pixel is proportional to the accumulated value of the light. Of these two methods, the ray tracing method is more suitable for this subject. First, the performance requirements of the projection method grating system are very high; second, the accumulated value of the projection method is limited by the color depth of the shading system; so, it will affect the display accuracy; third, the projection method does not support forward display, while the ray tracing method supports forward display, which can take into account image quality and calculation speed. Through analysis and comparison, the author uses the method of ray tracing.

RETRACTED

#### 3.5.2. Ray Tracing Algorithms

*(1) Principle of Ray Tracing Algorithm*. Ray tracing is a multifunctional technique, which can use the same model to simulate the specular reflection and refraction of the light source and the ambient incident light on the surface and realize the scene blanking and generate shadows, etc. [18]. The ray tracing algorithm is an important algorithm for generating photorealistic graphics and can also be used as a basic technology for volume rendering.

The method of generating the DRR image is as follows: first, the ray tracing method needs to set up a light source, emit light from the light source to the 3D model, and set up a receiving plane at the same time. Then, watch the light coming from the light source, if the ray does not intersect the model, the ray will exit the frame and the trace will end. These rays are not the focus of the study. If the light intersects the scene in the scene, it must be divided into the following situations:

1. The object where the intersection is located is an opaque object, the surface is an ideal diffuse reflection surface, and the ray tracing ends
2. The object where the intersection is located is an opaque object, the surface is an ideal mirror reflection surface, and the light continues to trace along the direction of the mirror reflection
3. The object where the intersection is located is a transparent or semitransparent object, and the light continues to trace along its regular transmission direction according to the laws of reflection and refraction

Finally, when the ray intersects the receiving plane, the attenuation value of the ray is recorded to complete the tracing of the ray.

Since the ray tracing method needs to trace each ray from the viewpoint, it must involve a large number of intersection operations between the rays and the three-dimensional model. In order to make the ray tracing algorithm practical, it is necessary to improve the efficiency of the intersection operation and simplify the calculation.

*(2) Implementation of Ray Tracing Algorithm*. The implementation method of the simplified ray tracing algorithm is as follows: a virtual parallel X-ray is passed through the three-dimensional model established based on the CT image data, and the starting point of the ray is equivalent to the X light source. The attenuation of the ray is calculated from the CT value of the voxel that the ray intersects. The CT value is related to the density of the three-dimensional model; so, the attenuation value of the light can be calculated by using the CT value. Compute each voxel that intersects this ray, up to the 3D model. From these accumulated values, a pseudovisible optical density value for display can be calculated and then displayed on the screen like an X-ray image.

RETRACTED

### 3.6. Overview of Image Registration

#### 3.6.1. The Principle and Implementation of Image Registration

The registration of medical images is to use image registration technology to calculate the spatial transformation relationship between two images, so that the points in the floating image are spatially consistent with the corresponding points on the reference image after the transformation; that is, the same anatomical point on the human body has the same spatial position on the two medical images. Simply put, one of the images is selected as the reference image (ReferenceImage) to be fixed, and the floating image (FloatingImage) is spatially transformed so that the points on the same position of the two images correspond to the same anatomical position [19]. The ideal registration result is that all the medically valuable feature points in the two images can be in one-to-one correspondence [20].

The medical image registration method consists of four parts: feature space (FeatureSpace), search space (SearchSpace), search algorithm (searchalgorithm), and similarity measure (SimilarityMeasure). Feature space refers to the distribution of feature information in images to be registered. The search space refers to the range of spatial transformation of the floating image [21]. The search algorithm refers to the method of calculating the spatial transformation of the floating image, that is, the method of finding the optimal transformation matrix parameters [22]. Similarity measures refer to quantitative metrics used to measure the quality of image registration. The process of medical image registration is shown in Figure 3.

## 4. Results and Discussion

According to the change of the key parameter *X* value, the mutual information value in different situations can be obtained. Taking the *X* value as the *X* axis and the mutual information value as the *Y* axis, according to the corresponding relationship, the second-order curve fitting function can be used to fit the change curve of mutual information [23].

Positive mutual information value fitting curve: the positive mutual information value fitting curve obtained during the research period is shown in Figure 4; in this fitting curve, the mutual information curve has two extreme values [24].

RETRACTED

Lateral fitting curve was as follows: the lateral fitting curve of the CT image processing results of the patient is shown in Figure 5; as explained in the figure, the lateral fitting curve only contains one extreme value [25].

Accuracy is as follows: the number of accurate cases in this research method is 77, with an accuracy rate of 96.3%.

## 5. Conclusion

The authors propose a method for sports medicine image modeling and injury prevention during sports training. The research of the specific content of this method is based on the principle of two-dimensional and three-dimensional registration; during the research, the program is written strictly according to the registration principle, and the correctness of this method is effectively tested by means of experimental methods. Digital image reconstruction measures based on 3D models can be based on ray tracing methods. The related parameter optimization method is the simulated annealing method. According to the research situation of medical image 3D modeling and registration technology for precision radiotherapy device, the functions of medical image navigation system can be enriched to enhance the accuracy of the model. In order to shorten the modeling time, the complexity of 3D modeling can also be appropriately reduced according to the actual situation of the research work. According to the real-time requirements of registration during surgery, the reconstruction speed can also be improved on the basis of improving the digital image reconstruction algorithm. To sum up, the 3D modeling and registration technology of medical images for precise radiotherapy devices plays an important role in the field of clinical diagnosis.

## Figures and Tables

**Figure 1:** DICOM data set structure.

**Figure 2:** Schematic diagram of visualization pipeline.

**Figure 3:** Schematic diagram of medical image registration process (high-end).

**Figure 4:** Positive fitting curve.

**Figure 5:** Lateral fitting curve.

**Table 1:** Time spent on a single image of each noise filtering method (unit: s).

Noise filtering method	Median filter	Average neighbor filtering	Gaussian low-pass filtering
Processing time	0.4992	0.0312	0.2184

## Data Availability

The data used to support the findings of this study are available from the corresponding author upon request.
